# An extraordinary T/NK lymphoma, nasal type, occurring primarily in the prostate gland with unusual CD30 positivity: case report and review of the literature

**DOI:** 10.1186/1746-1596-8-94

**Published:** 2013-06-17

**Authors:** QingPing Jiang, Shaoyan Liu, Juan Peng, Hanzhen Xiong, ZhongTang Xiong, Yuexin Yang, Xuexian Tan, Xingcheng Gao

**Affiliations:** 1 Department of Pathology, The Third Affiliated Hospital, Guangzhou Medical University, Guangzhou 510150, China; 2 Department of Urology, The Third Affiliated Hospital, Guangzhou Medical University, Guangzhou 510150, China

**Keywords:** Prostate, Extranodal NK/T cell lymphoma, Nasal type, CD30, T-cell receptor genes, Lymphoepithelial lesion

## Abstract

Extranodal NK/T cell lymphoma(NKTCL), nasal type, occurring primarily in the prostate gland, is extremely rare. We present a case of primarily prostatic NKTCL in a 59-year-old man suffering from dysuria. Histological examinations revealed that diffused, large-sized, pleomorphic lymphocytes were arranged in an angiocentric distribution with large areas of geographic necroses. Additionally, the prostatic glands were diffusely infiltrated by heteromorphous lymphocytes forming lymphoepithelial lesions. The tumor cells were strongly expressed CD3ϵ, CD56, TIA-1, granzyme B and EBV-encoded RNAs. And interestingly, the lymphoid cells were also strongly immunoreactive with CD30. A rearrangement study showed T-cell receptor γ-chain gene rearrangement with monoclonal appearance. Though postoperative combination of chemotherapy was given, the patient died four months later. Our observation and other literatures indicate that extremely rare NKTCLs unusually express CD30. TCR gene rearrangement existed in some NKTCL, suggesting that a subset of NKTCL may be a mixed NK/T-cell differentiation.

**Virtual slides:**

The virtual slide(s) for this article can be found here: http://www.diagnosticpathology.diagnomx.eu/vs/9671878568932824.

## Introduction

Extranodal NK/T cell lymphoma, nasal type (NKTCL) is well known as an aggressive tumor that is characterized by vascular damage and destruction, prominent geographic necrosis, and associated with Epstein-Barr Virus (EBV). The most common sites involve the upper aerodigestive tract, with the nasal cavity being the prototypic site. The extranasal sites that NKTCL favors include skin, gastrointestinal tract, and soft tissues [1,2]. The NKTCL involving prostate is very rare [3]. Primary NKTCL has been not reported. Here, we report a case of primary prostate NKTCL in a 59-year-old man with CD30 positive expression and T-cell receptor γ-chain gene rearrangement.

## Case report

### Clinical history

A 59-year-old man suffered from low fever for one month, increased frequency of urination and dysuria for approximately a week. A computed tomography (CT) scan revealed benign hyperplasia in the prostrate. Therefore, a routine procedure of transurethral resection of prostate was conducted. After the diagnosis of NKTCL, since there was a great possibility of dissemination of other sites’ NKTCL, the patient was referred to a whole body positron emission tomography/computed tomography (PET/CT) study to search for a potential primary tumor, but no other abnormality was found. The lesion was proved primarily occurred in prostate and just in stageI. However, despite three courses of chemotherapy were given, the patient died after four months with wide dissemination of the tumor and rapidly deteriorated clinical symptoms.

## Materials and methods

Tissues were routinely fixed in 10% neutral buffered formalin and embedded in paraffin. Three micrometer-thick sections were stained with hematoxylin and eosin. Immunohistochemical analyses were performed using the ChemMate Envision/HRP Kit (Dako, Glostrup, Denmark). Antibodies used in this study were CK, PSA, PSAP, P504S, Vimentin, LCA, CD2, CD3ϵ, CD7, CD4, CD8, CD56, CD30, ALK, TIA-1, granzyme-B, CD20, CD79a, CD138, CD68, TdT, and ki-67. The antibodies were obtained from Dako Cytomation (Carpinteria, CA) and Santa Cruz Biotechnology (Santa Cruz, CA). Slides were dewaxed and rehydrated routinely and then were treated with 10 mmol citrate buffer (pH 6.0) in a microwave for antigen retrieval. After incubation with diluted primary antibodies, slides were treated with the ChemMate Envision/HRP Kit for 30 minutes at room temperature followed by development with diaminobenzidine (DAB) for visualization.

In situ hybridization(ISH) was performed to detect the Epstein-Barr virus encoded RNAs(EBERs) (DIG-AP, A300 K.9901; PanPath, Netherlands). Detection process was conducted according to manufacturer’s instructions.

For cytogenetic analysis, the paraffin tissue DNA was prepared with a tissue DNA extraction and purification kit (Dneasy TM Tissue Kit, Qiagene, CA). T-cell receptor rearrangement studies were performed. Two sets of primers (tube A, 145–255 bp; tube B, 80-220bp) were used to amplify the rearranged T-cell receptor (TCR)-γ gene. A T cell lymphoma case with a known monoclonal rearrangement was used as a positive control, a non-lymphoid and hematopoietic tumor was used as a negative control, and a reaction without template DNA was simultaneously run as a blank control. β-actin was amplified as an internal control. The detection process was conducted by methods described previously [4].

### Pathological findings

The microscopic findings of the prostate revealed the lesion was mainly infiltrated by intermediate- to large-sized tumor cells with angiocentric and angiodestructive growth pattern. The prostate gland damage was also noted in the lesion. The tumor cells had irregular or oval, hyperchromatic nuclei with one to several prominent nucleoli, accompanying notable pathological mitosis and apoptosis (Figure 1a-f). The tumor cells expressed LCA, CD3ϵ, CD2, CD7, CD30, and CD56, perforin, TIA-1, rather than CK, PSA, PSAP, P504S, Vimentin, CD79a, CD20, CD4, CD8, and ALK (Figure 2). Ki67 was expressed in nearly 90% of the tumor cells. EBERs signals were detected diffusely in nuclei of the tumor cells (Figure 3). Based on these results, the diagnosis of NKTCL with CD30 expression was made. The rearrangement study showed TCRG gene rearrangement with monoclonal appearance (Figure 4).

**Figure 1:** **Histological examination.** (**a**) Under low magnification, the tumor diffuses with the large areas of necrosis (H&E staining, original magnification × 2). (**b**) The normal areas of prostate near the tumor (H&E staining, original magnification × 4). (**c**) Tumor cells invade vessel wall seriously (H&E staining. original magnification × 20). (**d**) Glands are destroyed by tumor cells (H&E staining. Original magnification × 20). (**e**, **f**) The tumor cells were large with one to several prominent nucleoli, accompanying notable pathological mitosis and apoptosis (H&E staining. Original magnification × 40).

**Figure 2:** **Immunohistochemical results.** (**a**) Remnant gland epithelial cells were positive for CK (SP, original magnification × 40). (**b**) LCA positive expression for tumor cells (SP, original magnification × 40). (**c-e**) Tumor cells were positive for CD3, CD2 and CD56, respectively (SP, original magnification × 40). (**f**) Tumor cells were positive for CD30 (SP, original magnification × 40).

**Figure 3:** EBERs positive expression in tumor cells (→) (ISH, original magnification × 40).

**Figure 4:** **Multiplex PCR for T-cell receptor c-chain gene using 6% polypropylene gel electrophoresis.***Lane 1*, DNA Marker. *Lane 2* monoclonal(positive) control of tube A. *Lane 3* polyclonal(negative) control of tube A. *Lane 4* blank control of tube A. *Lane 5* monoclonal T-cell receptor c-chain gene rearrangement in reproducible duplicate of tube A. *Lane 6* monoclonal(positive) control of tube B. *Lane 7* polyclonal(negative) control of tube B. *Lane 8* blank control of tube B. *Lane 9* monoclonal T-cell receptor c-chain gene rearrangement in reproducible duplicate of tube B. *Lane 10* β-actin.

## Discussion

Besides of prostatic adenocarcinoma, there are a few other types of neoplasms occurring in prostate which are difficult to determine their primary origins, such as prostatic squamous carcinoma [5]. Lymphomas of prostate, either primary or secondary, are very rare. The types are mainly consisted of B-cell lymphomas [6], including diffuse large B-cell non-Hodgkin’s lymphoma (DLBL) [7], mucosa-associated lymphoid tissue (MALT) lymphoma [8], and mantle cell lymphomas [9]. Only three cases of T-cell lymphomas involving the prostate have been reported, but none of them was primary [10,11]. According to the criteria of Bostwick [3], primary prostatic lymphoma could be diagnosed subject to the fulfillment of the following conditions: primary symptoms are attributed to prostatic enlargement; the disease is almost localized to the prostate; and, NKTCL diagnosis does not include lymph nodes, liver, spleen and other organs in 1-month. The symptoms of the present case were only associated with prostatic hyperplasia, and no tumor was detected in other organs through the systemic PET-CT detection. In this manner, the primary lymphoma of prostate was confirmed. The tumor showed typical angiocentric and angiodestructive growth patten, a typical immunophenotype expressing CD56, CD3ϵand EBERs positive detection with ISH. Collectively, the lesion was best recognized as NKTCL.

Cell morphology of NKTCL is comprehensive. Most cases comprise middle cells mixed a few small- and large-sized cells, and usually do not have nucleoli. The present case is mainly composed of large or anaplastic cells containing several nucleoli. This tissue change may indicate a poor prognosis [2]. Expression of CD30, an important marker for anaplastic large-cell lymphomas, in NKTCL is rare. One case of CD30+ NKTCL occurring on skin was reported in 2008 [12]. In that case, Strong CD30, CD3ϵand CD56 immunoreactivities were noted in large atypical mononuclear cells. That patient died within 8 months after the onset of skin lesions. In another report, fine-needle aspiration of an large adrenal mass and CSF cytology showed that large atypical cells were positive for CD30, CD43, and CD56. The patient also died a few days after the final diagnosis was achieved though with high dose intravenous dexamethasone [13]. The case in the present study also revealed diffusely CD30 expression in large tumor cells. According to these cases, it is speculated that NKTCL with large cells can express CD30 and indicate a worse prognosis. But more cases are necessary to prove it. In 2013, 17/40 cases CD30-positive were found in a report of 73 cases at MD Anderson cancer center, but had no further discussion about clinical threatment and prognosis [14].

The rearrangement TCR genes is an important supplement to the diagnosis of T-cell non-Hodgkin lymphoma. TCR genes are clonally rearranged in most cases of PTCL, NOS [15], while only a small proportion of NKTCLs show clonal rearrangement [16,17]. However, some studies identified monoclonal TCRG gene rearrangement in a significantly higher proportion of NKTCLs, suggesting a mixed NK/T-cell differentiation in a subset of these tumors [18,19]. The present case maybe belong in this subset.

Though with characteristic microscopic finds and Immunohistochemical expression, differential diagnosis is requisite before making a definite NKTCL, since prostatic NKTCL is so rare. Poorly differentiated carcinoma with diffuse tumor cells might represent some histological similarity with NKTCL, but it usually dose not display angiocentric distribution with large geographic necroses and lymphoepithelial lesions, and it often can be found some heteromorphic glands. Immunohistochemical results show expression of epithelial markers such as CK, CK8/18 and PSA et al., rather than lymphocyte ones. Another rare tumor, prostatic stromal sarcoma, is often showed pervasive small and medium-sized round cells around the residual glands too [20]. It is suspiciously derived from mesenchymal pluripotent stem cells in the prostatic stroma and usually express CD10, CD34 and PR.

## Conclusion

The case reported the possibility of NK/T cell lymphoma primarily occurring in prostate. Compared with that of other organs, the prognosis of the prostate disease is also poor. The prognoses of those tumors mainly comprised of big cells with CD30 positive expression are quite unclear because of rare cases. The rearrangement of TCR genes in NKTCL suggests a mixed NK/T-cell differentiation in a subset of these tumors.

### The medical/scientific value of this case report

It is well known the prognosis of prostatic adenocarcinoma depend on its Gleason score, positive surgical margin(PSM), perineural invasion (PNI), and abnormal expression of some genes [21,22]. Nevertheless, these items are not fit with other less happened neoplasms in prostate, such as lymphoma. Though the primarily prostatic NKTCL is very rare, its accurate diagnosis is medically significant because it is highly aggressive and its clinical prognosis is as poor as ones in other sites. Its treatment is supposed to take chemical therapy as done as NKTCL of other organs, instead of traditional androgen deprivation therapy for prostatic carcinomas. Usually, diagnosis procedure for a primarily prostatic CD30 positive NKTCL includes the following steps: 1. H&E staining reveals diffuse infiltrated large-sized or anaplastic tumor cells with remarkable apoptosis and angiocentric necrosis; 2. Immunohistochemical results present the expression of LCA, CD2, CD3ϵ and CD56, perforin, TIA-1, and CD30; 3. EBERs are detected in tumor cells. 4. No tumor was detected in other organs.

## Consent

To publish this case report and accompanying images, written informed consent was obtained from the patient’s family.

## Abbreviation

NKTCL: Natural killer/T cell lymphoma.

## Competing interests

The authors declare that they have no competing interests.

## Authors’ contributions

QP J drafted the manuscript and participated in the final diagnosis. ZT X conducted the gross examination and final diagnosis. SY L conducted the immunohistochemical study. YX Y participated in the immunohistochemical study. J P and HZ X participated in the final diagnosis. XC G revised manuscript critically for important intellectual content and had given final approval of the version to be published. The final manuscript was read and approved by all authors.
